# Enhancers and chromatin structures: regulatory hubs in gene expression and diseases

**DOI:** 10.1042/BSR20160183

**Published:** 2017-04-28

**Authors:** Zhenhua Hu, Wee-Wei Tee

**Affiliations:** 1 Institute of Molecular and Cell Biology, A*STAR, 61 Biopolis Drive, Proteos 138673, Singapore; 2 Department of Physiology, Yong Loo Lin School of Medicine, National University of Singapore, Singapore 117597, Singapore

**Keywords:** chromatin, DNA looping, Enhancers, gene expression

## Abstract

Gene expression requires successful communication between enhancer and promoter regions, whose activities are regulated by a variety of factors and associated with distinct chromatin structures; in addition, functionally related genes and their regulatory repertoire tend to be arranged in the same subchromosomal regulatory domains. In this review, we discuss the importance of enhancers, especially clusters of enhancers (such as super-enhancers), as key regulatory hubs to integrate environmental cues and encode spatiotemporal instructions for genome expression, which are critical for a variety of biological processes governing mammalian development. Furthermore, we emphasize that the enhancer–promoter interaction landscape provides a critical context to understand the aetiologies and mechanisms behind numerous complex human diseases and provides new avenues for effective transcription-based interventions.

## Introduction

Mammalian development and tissue specificity originate from the tightly controlled hierarchy of gene expression events [1–3]. Gene transcription starts with regulatory events at promoters, where transcription factors (TFs) bind to *cis*-regulatory sequences at core promoters immediately upstream of transcription start sites (TSSs) and promote the assembly of the RNA polymerase II (RNAPII) transcription preinitiation complex, assisted by general TFs (GTFs) and co-activators (Figure 1A) [4,5]. RNAPII is paused around the TSSs after nascent RNA of approximately 50 bp has been transcribed, and extra signals are required for subsequent RNAPII escape into effective elongation along the gene body. In addition to these promoter-proximal events, gene expression is also dependent on the inputs from distal *cis*-regulatory elements, including enhancers and insulators. Enhancers are of particular interest as they tend to be active in a cell type specific manner whereas promoters are apparently more ubiquitously used [6–8]. Notably, enhancers can act at long distances away from the TSSs and independent of their orientation [9]. Studies have shown that enhancers can potentially influence different steps of the transcription cycle, from RNAPII recruitment, promoter-proximal pause-release, to transcription elongation, underscoring the importance of these regulatory DNA elements in the control of gene expression [9].

**Figure 1:** Enhancers act as regulatory hubs in gene activation (**A**) Gene activation requires the co-ordinated actions of multiple factors and processes. One of the key processes involved is the cognate enhancer–promoter interaction mediated by TFs and many other cofactors, including mediator/cohesin complexes and chromatin regulators. Transcribed enhancer RNAs (eRNAs) from active enhancers in turn regulate different stages of transcription, including enhancer–promoter looping and the release of paused RNAPII. Typically, gene transcription is associated with distinct chromatin structures, such as the enrichment of histone H3 lysine 27 acetylation (H3K27ac) and histone H3 lysine 4 monomethylation (H3K4me1) at enhancers, histone H3 lysine 4 trimethylation (H3K4me3) at promoters and histone H3 lysine 36 trimethylation (H3K36me3) at gene bodies. (**B**) Clusters of TF binding sites (TFBSs) at enhancers, including super-enhancers, serve as regulatory hubs to synthesize information from multiple sources of stimuli. Biologically important TFs, including signalling terminal effectors, often associate with each other and bind to (super-)enhancers. Super-enhancers tend to show stronger enhancer activity than typical enhancers.

Enhancers are largely responsible for shaping cell type-specific gene expression programmes through successful and specific communication with their cognate gene promoters. For enhancers to exert their regulatory functions at the right time and right place, three requirements have to be satisfied: (i) enhancers should be accessible, which requires the genome to adopt appropriate local chromatin structure to expose TF binding motifs at enhancers; (ii) enhancers and promoters have to interact in a cognate fashion, which requires the genome to adopt appropriate higher order chromatin structure, so that enhancers and target promoters are placed in physical proximity and importantly, (iii) both local chromatin accessibility and higher order chromatin organization have to be compatible with different cell types and developmental stages. In this review, we first briefly introduce the role of enhancers in gene expression, followed by the chromatin structural features associated with the regulation of enhancer accessibility and activity. We will also summarize the mechanisms that guarantee the specificity of enhancer–promoter interactions required for cell type and developmental stage-specific gene expression. We then conclude with the notion that the spatial clustering of enhancers may serve as regulatory hubs to coalesce and synthesize information arising from the dynamic interactions between TF binding, signalling effectors and chromatin environment and emphasize the importance of integrating and interpreting different types of ‘omics’ data in the context of enhancer–promoter interactions.

## Expanding roles of enhancers in gene transcription

Enhancers were first discovered in the SV40, whose genome contained several elements that hugely increased the expression of the rabbit β-globin gene in a position-, orientation- and distance-independent manner [10–12]. This finding has since inspired intensive research on how enhancers regulate gene transcription over a range of distances, which may be as long as one megabase or beyond [13]. Classically, enhancers were thought to promote gene transcription by facilitating the establishment of cognate enhancer–promoter interactions and promoting RNAPII loading at promoters; however, the detection of RNAPII-transcribed extragenic non-coding eRNAs suggests that enhancers are functional transcriptional units [9,14,15], a property that was previously considered to be exclusive to promoters. Moreover, enhancer transcription also occurs in a cell type- and/or context-specific manner, involving specific TF binding that functions to maintain enhancer accessibility, potentiating downstream assembly of the RNAPII apparatus [9,16,17]. Though some studies have suggested that eRNAs might be a by-product due to the high concentration of RNAPII at enhancer–promoter interaction foci [9,18]. Other reports show that eRNAs can actively promote gene activation by reinforcing enhancer–promoter looping and stability [19,20], as well as promoting the release of paused RNAPII at promoters by interfering with the negative elongation factor (NELF) complex (Figure 1A) [21]. Notably, similar to other non-coding RNAs, eRNAs can also interact with selective TFs and chromatin regulators to augment their binding to key regulatory DNA regions [9,22]. Interestingly, a recent study showed that eRNAs can directly interact with histone acetyltransferases CREB binding protein (CBP), that contributes to the permissive local enhancer chromatin structure, driving target gene expression [23]. Importantly, knockdown of eRNAs as well as programmable recruitment of eRNAs to specific enhancer elements have provided strong support for a functional role of eRNAs *in vivo* [9,18,20,22,24–26]. However, we also caution against a generalized instructive model of eRNAs in directing gene expression changes. The very act of enhancer transcription by RNAPII may also direct chromatin changes at enhancers, independent of eRNA transcripts [27]. Taken together, these findings present an updated view of how eRNAs, as well as the act of enhancer transcription, can promote gene activation via multiple mechanisms, acting at all levels of the transcription cycle. Understanding the hierarchy of events and the players involved during enhancer–promoter DNA looping may reveal further insights into how enhancers operate in relation to promoter events. While the general consensus is that enhancer events precede promoter activity, with abundance of studies showing that deletion of enhancer elements affect promoter activity, it is noteworthy to mention that exceptions do exist. For example, Kim et al. [14], showed that although the binding of RNAPII to the arc enhancer is independent of the arc promoter, the transcription of eRNAs is apparently dependent on the formation of enhancer–promoter interaction. This argues against a requisite need for eRNAs in chromatin looping, a finding also reported by Hah et al. [28], showing that inhibiting eRNA transcription does not appear to affect enhancer–promoter looping at least under the selective conditions tested. Experiments directed at identifying protein complexes at enhancers and promoters coupled with the ability to manipulate loop formation may help illuminate the order of events underlying enhancer–promoter communications. In this regard, the recent identification of the Integrator complex as a key regulator of enhancer function is an important finding [17]. Integrator can be recruited to enhancers in a signal-dependent manner and is required for both the induction and maturation of eRNAs. Importantly, depletion of Integrator abrogates stimulus-induced enhancer–promoter chromatin looping. Although Integrator is also present at promoters, it apparently exerts a different function.

## Enhancer activities and chromatin structure

Genome wide census studies have been carried out to catalogue functional enhancers across different cell types and species, including human and mouse. These studies revealed that the number of enhancers is far more than that of protein-coding genes, suggesting that a gene might be under the regulation of multiple enhancers and can respond to different signals of varying strengths by the differential usage of a subset of enhancers [1,29–32]. In particular, the generation of chromatin state maps have led to the identification of distinctive chromatin features that define three different enhancer states: active enhancers are typically marked by H3K27ac and H3K4me1, whereas silent enhancers are typically enriched for histone H3 lysine 27 trimethylation (H3K27me3) [33,34]. Interestingly, the third class of enhancers is enriched for both repressive H3K27me3 and active H3K4me1 modifications; these enhancers have been termed ‘poised’ enhancers and are associated with developmental genes that are lowly expressed in embryonic stem cells (ESCs) but poised for activation when differentiation signals are present [34–37]. Upon ESC differentiation, many of these poised enhancers transit to an active enhancer state concomitant with developmental gene activation, whereas other active/poised enhancers associated with ESC self-renewal maintenance will be decommissioned through the loss of H3K4me1 [38].

Further to the presence of H3K4me1 and H3K27ac, active enhancers exhibit higher sensitivity to DNase I digestion, indicative of increased chromatin accessibility [8]. Notably, these DNase I hypersensitive regions tend to be enriched for histone variants H2A.Z and H3.3, known to facilitate transcription activation through higher nucleosome turnover [39–41]. Therefore, the rewiring of chromatin accessibility is the key to differential enhancer usage and activity during development. For example, the differentiation and maturation of cerebellar granule neurons (CGNs) in developing mice is accompanied by substantial changes in the landscape of DNase I hypersensitive sites (DHSs) that are enriched for CGN-specific enhancers [42].

## Regulation of enhancer accessibility by chromatin structure and TFs

The nucleosome is the basic repeating unit of chromatin structure [43]. As DNA is wrapped around the nucleosome, transcription regulatory elements may be occluded; this reduced accessibility must be alleviated to allow unimpeded access of TFs, RNAPII and other transcriptional machinery to the underlying DNA sequence. Extensive chromatin remodelling is thus intimately tied to enhancer activity and as a consequence, the variable and dynamic accessibility of enhancers provide an important mechanism behind gene expression plasticity and response to environmental cues. To illustrate this, widespread changes in enhancer chromatin accessibility have been observed during cerebellar development, in a manner that correlates with the binding of zinc finger in cerebellum (ZIC) 2, a key forebrain TF [42].

Several ATP-dependent chromatin remodellers have been implicated in enhancer function [44,45]. For example, Brg1, a subunit of the BAF chromatin remodelling complex, specifies B-cell’s fate by facilitating the access of lineage-specific TFs to their enhancers through nucleosome displacement in lymphoid progenitor cells [46]. On the other hand, E1A-binding protein P400 (EP400), a SWR1 class chromatin remodelling protein, activates gene transcription by depositing H2A.Z and H3.3 in enhancers and promoters [47]. Last but not the least, chromodomain helicase DNA-binding domain 7 (CHD7), a chromatin remodelling enzyme from the CHD family, co-operates with p300 co-activator and ESC master TFs octamer-binding TF 4 (OCT4), SRY (sex-determining region Y)-box 2 (SOX2) and NANOG (OSN (OCT4, SOX2 and NANOG)) at enhancers to control ESC cell identity [6,48,49].

Further to the chromatin remodellers, TFs themselves can affect nucleosome dynamics. For example, through co-operative binding, different TFs can efficiently bind to nucleosome-embedded motifs, whereas they can only bind weakly if alone [50]. TFs can also interact with chromatin remodelling factors to trigger an assisted loading mechanism, where the initial association of one TF with its TFBSs can recruit chromatin regulators to remodel locally closed chromatin, priming the later binding of secondary TFs and triggering a positive feedback mechanism [31,44,51].

Of particular relevance to this discussion is the class of pioneer TFs. Pioneer factors are a special type of TFs that have strong DNA-binding activity. However, unlike most other TFs, they are able to gain access to silent genes that are devoid of histone modifications but instead enriched for linker histones that compact the chromatin. Mechanistically, pioneer TFs are able to recognize fully or partially exposed motifs on the nucleosome surface and upon engagement, can displace linker histones, inducing an open chromatin region to enhance the binding of other TFs and the assembly of transcriptional complexes [52–54]. This is best illustrated in the case of forkhead box A1 (FoxA1), a classical pioneer TF involved in endoderm specification [52,54]. The crystal structure of FoxA1 revealed a DNA-binding domain (DBD) that shares high similarity with that of linker histones, as well as a C-terminal domain which binds to core histones. The DBD is able to contact the FoxA DNA motif present on one side of the DNA helix, while leaving the other side of the helix open for histone binding. On the other hand, the C-terminal domain of FoxA1 binds directly to core histones, thereby disrupting the interaction between nearby nucleosomes [54–57]. This unique property of pioneer factors makes them ideal regulators of enhancer remodelling. In the case of FoxA TFs, they play a critical role in maintaining chromatin accessibility at liver-specific enhancers, potentiating the recruitment of other liver-specific TFs such as HNFa to activate the liver gene expression programme [16].

Importantly, pioneer factors can assist the binding of other TFs to inaccessible target regions, including enhancers. For example, c-Myc, a key TF involved in various cellular processes including nuclear reprogramming, is unable to bind to closed chromatin targets. However by partnering with the pioneer factors OCT4 and SOX2, it can acquire pioneer activity and bind to the degenerate E-box motif on nucleosomes, promoting the activation of stem cell related genes during the reprogramming process [53,58]. In this regard, it is noteworthy that many of these pioneer TFs, such as OCT4, SOX2 and FOXA, are key master regulators of cell fate that act high in the hierarchy of gene regulatory networks [52,53].

Interestingly, sequence analysis reveals that many DNA regulatory elements, including enhancers, have high intrinsic nucleosome occupancy [59,60]. Although nucleosomes generally constitute barriers to TF binding, pioneer TFs may exploit this increased nucleosome occupation to facilitate their binding on enhancers. Given that enhancer remodelling often precedes promoter gene activity [61,62] and unlike promoters, enhancers tend to become open in a tissue-specific manner [8]. An interesting proposition is that higher nucleosome occupancy at enhancer regions may serve as a protective mechanism against unintended TF-enhancer interactions; it may be that by limiting enhancer access to a small but privileged group of pioneer TFs, tighter control on tissue-specific gene expression may be achieved [52].

## Compartmentalization of the three-dimensional genome shapes the enhancer–promoter interaction landscape

Enhancer–promoter DNA loops represent interactions that are embedded in larger genomic compartments. Genome organization happens at different levels, ranging from the primary level of organization that generates arrays of nucleosomes, which are further compacted into chromatin fibres, to the higher levels that determine the overall 3D organization of the genome in the nucleus [63]. This higher-order organization is necessary as the length of the eukaryotic genome is orders of magnitude longer than the diameter of the nucleus and hence must be efficiently compacted. However, the multiple levels of higher-order chromatin folding will invariably create contacts among genomic loci, such as enhancer-harbouring regions. Clearly, mechanisms must be in place to ensure that enhancers only interact with their cognate promoters, and also to prevent interactions between enhancers and promoters that are incompatible with cellular functions. In the following two sections, we summarize the current understanding of the specificity of interactions mainly achieved by compartmentalizing and insulating the genome into discrete regulatory domains, termed as topologically associating domains (TADs) [64–66].

## Inter-TAD interactions are inhibited by TAD borders and architectural proteins

Investigations utilizing a series of chromatin conformation capture techniques have showed convincingly that chromosomes are organized in TAD units, which are usually megabase sized discrete genomic regions that feature frequent local intra-TAD chromatin interactions (for example, enhancer–promoter loops) (Figure 2A) [67–73]. TADs are separated by TAD borders and inter-TAD interaction frequency is very low [67,74]; however, the strength of TAD borders in separating TADs may vary, giving rise to differential ratios of intra-TAD to inter-TAD interactions [75]. There is evidence suggesting that the inhibitory effects of TAD borders are largely mediated by architectural proteins, including CCCTC-binding factor (CTCF) and cohesin complexes [67,76–78], and that the depletion of these architectural complexes could result in decreased intra-TAD and increased inter-TAD interactions [79–81].

**Figure 2:** Disorganization of TADs is associated with aberrant phenotypes (**A**) A schematic representation of TAD organization. TADs are separated from each other by TAD borders bound by architectural proteins such as CTCF. Genomic interactions, such as that between cognate enhancers and promoters, are constrained within a TAD (intra-TAD interaction), while inter-TAD interactions are generally inhibited. (**B**) *De novo* formation of a TAD, followed by a gene duplication event, aberrantly juxtaposes the potassium voltage-gated channel subfamily J member 2 (*KCNJ2*) gene and an ectopic regulatory region within the same TAD, resulting in Cooks syndrome. (**C**) TAD disruptions are associated with limb abnormalities. An extra TAD, due to the genomic duplication of the *IHH* locus and its associated TAD border (blue), leads to polydactyly. In contrast, brachydactyly is caused by a genomic deletion across the TAD border separating the *EPHA4* and *PAX3* loci (red and green respectively), resulting in the dysregulation of *PAX3* by an ectopic *EPHA4* enhancer. Finally, a genomic inversion involving *IHH* locus (blue) and its neighbouring TAD (red) exposes *IHH* to toxic regulation by an *EPHA4* enhancer, leading to F-syndrome.

Organizing the genome into discrete TADs has important biological consequences. For example, cell identity genes and lineage-specific developmental genes are arranged in TADs that are insulated from each other in ESCs. Such organization helps to facilitate the co-ordinated activation of cell identity genes and repression of developmental genes, which is crucial to the maintenance of self-renewal and pluripotency [49,82]. In addition, a promoter and its regulatory pool of enhancers also tend to reside in the same TAD, such as the cystic fibrosis transmembrane conductance regulator (*CFTR*) gene, whose expression is regulated by multiple enhancers located within the same TAD [83]. However, it should also be pointed out that TAD borders are not rigid and that TAD organization can be altered in response to environmental stimuli. This is primarily driven by the redistribution of architectural proteins and leads to a decrease in TAD border strength and an increase in inter-TAD interactions [84]. Furthermore, regulated cross-talk between TADs can occur, such as the merging of neighbouring TADs, as observed in the humoral immune response during B-cell maturation in germinal centres [85]. However, aberrant disruption of normal TAD organization risks exposing promoters to ectopic distal enhancers, resulting in undesirable phenotypes. For example, Franke et al. [86] found that the *de novo* formation of a TAD, followed by a gene duplication event, underlies the aetiology of Cooks syndrome (Figure 2B). In addition, altered TAD borders encompassing the *WNT6-IHH/EPHA4/PAX3* loci can lead to various human limb malformations, including brachydactyly, F-syndrome and polydactyly (Figure 2C) [87]. Further to these developmental disorders, disruption of TADs can lead to the dysregulation of tumour suppressors and oncogenes in cancer [88]. Cancers are characterized by increased genomic rearrangements and frequently acquire (epi)genetic changes. These factors can directly affect TAD function. For example, a chromosome 3 inversion event recently described in acute myeloid leukaemia (AML) demonstrates how an inter-TAD relocation of an enhancer can ectopically activate the ecotropic viral integration site 1 (*EVI1*) oncogene [89]. Moreover, mutations in CTCF and cohesin complexes and the alterations in their binding sites have also been found in various cancers [90–92] and in some cases, perturbation of TAD boundary was sufficient to activate pro-oncogenes in non-malignant cells [92]. These findings point to a role of TAD in oncogenesis. Last but not the least, changes in the epigenome can also affect TAD function, as exemplified in *IDH*-mutant glioma where aberrant DNA methylation of CTCF-binding sites led to a partial disruption of TAD boundary formation [93]. Taken together, these studies highlight the profound affect of 3D genome organization on development and disease.

## Intra-TAD interactions are promoted by TFs and cofactors

While inter-TAD separation provides an efficient way to insulate genes from functionally toxic enhancers, intra-TAD DNA looping at the submegabase scale brings promoters and distal enhancers into physical proximity [94–97]. Unlike the 3D organization of TADs orchestrated by architectural proteins that are generally conserved and largely invariant across cell types and species [67], the enhancer–promoter interactome has to be dynamically regulated to be compatible with developmental stages and cell types. This is exemplified by recent studies showing that hundreds of novel enhancer–promoter interactions have been identified during human brain development [98], and that enhancer regions which interact with the *CFTR* promoter are different in different cell types [83]. This raises an important question: which factors are involved in enhancer–promoter interactions. Currently, enhancer–promoter interactions are thought to be mediated chiefly by cell type-specific TFs and co-activators and affected by local chromatin configurations [49,95–97].

An elegant demonstration of the role of TFs in enhancer–promoter interaction comes from a study of the TF specificity protein 1 (SP1) [97]. SP1 is known to mediate the long-range interaction between an interferon-β (IFN-β) enhancer and its promoter, which harbours an SP1-binding site. However, the ectopic insertion of SP1-binding sites on to heterologous promoters is able to force DNA looping of the IFN-β enhancer to the inserted binding sites, disrupting the original IFN-β enhancer–promoter interaction. Importantly, this event can occur independent of transcription, highlighting the instructive role of TFs in driving long-range interactions. In another example, oestrogen receptor α (ERα) has been shown to promote oestrogen-initiated transcription by mediating the long-range interactions between ERα enhancers and target promoters, a process that also involves several cofactors including AP-2γ and FoxA1 [99,100].

Some of the other key players involved in enhancer–promoter looping include the mediator and cohesin complexes [95]. Mediator is a large complex consisting of multiple subunits that interact with different TFs through different subunits, thereby specifying distinct enhancer–promoter interactions and cell-type specific gene expression [101]. For example, mediator subunit 1 (MED1) plays a critical role in shaping the interactions between OSN-bound enhancers and target genes that are important for the cell identity of ESCs [49,102]. In another notable example, in an effort to screen for regulators that affect the enhancer–promoter interaction and expression of *Oct4* in murine ESCs, Kagey et al. [95] identified a subset of mediator subunits and cohesin complexes in addition to other known TFs.

Many of the aforementioned factors, such as CTCF and MED1, physically bridge enhancer–promoter interactions. However, other players can affect enhancer–promoter interactions by regulating local chromatin structure. One such example is testis expressed 10 (TEX10), a key factor involved in the maintenance and establishment of pluripotency for ESCs [102]. With appropriate environmental cues, TEX10 is directed by NANOG to OSN enhancers, and facilitates the enhancers’ interactions with target promoters by recruiting the histone acetyltransferase p300 and the DNA demethylase Tet methylcytosine dioxygenase 1 (TET1) to create permissive chromatin structures that are H3K27ac enriched and DNA hypomethylated [102]. On the contrary, the expression of the N-methyl-D-aspartate (NMDA) glutamate receptor *GRIN2B*, a gene implicated in schizophrenia, is promoted by the interaction between *GRIN2B* promoter and its enhancer that is located 449 kb away; when SET domain bifurcated 1 (SETDB1)-mediated H3K9me3 is enriched around the TSS and bound by the repression-associated protein heterochromatin protein 1α (HP1α), a repressive chromatin structure is formed, leading to the disruption of enhancer–promoter interaction and subsequently *GRIN2B* inactivation [103–105].

## Enhancer clustering constitutes a signal-integration platform

We have so far discussed how an individual enhancer can contact its cognate promoter through the concerted action of architectural proteins and TFs. However, accumulating evidence shows that multiple TFBSs tend to cluster together at *cis*-regulatory regions (Figure 1B) [31]. For example, genome-wide analyses revealed that it is common for both enhancers and promoters to harbour multiple binding sites for the same TF [106,107]. Perhaps more interestingly, TFBSs for different TFs also tend to cluster together, constituting a highly dense binding platform, which can be as large as 12.5 kb [38,108]. These regulatory units have been termed as stretch enhancers or super-enhancers. Like typical enhancers, super-enhancers are enriched for H3K27ac with high H3K4me1 to H3K4me3 ratio and are sensitive to DNase I cleavage [8,109]. However, when compared with typical enhancers, super-enhancers tend to show higher enrichment for transcriptional co-activators such as MED1 and stronger enhancer activity (Figure 1B) [49,108,110–112]. Nevertheless, whether super-enhancers truly represent a novel transcriptional entity that is functionally different from typical enhancers that can act in isolation or additive, remains debatable [113]. A key question is whether the effect of super-enhancer as a whole is significantly larger than the sum of the effects of constituent enhancers. To clarify this, enhancer deletion type experiment is necessary to assess the relative contribution of individual enhancer compared with super-enhancer as a whole [114,115].

Notwithstanding the contentious mechanism of super-enhancers, the criteria used to define super-enhancers have proved to be extremely valuable in identifying key regulatory regions that are important for cell identity. Furthermore, it is clear that the clustering of enhancers for the same or multiple TFs provides functional importance for cellular functions. First, the clustering of submaximal TF recognition motifs and suboptimal spacing between the motifs might provide a strategy for the controlled balance between enhancer activity and specificity [116]. Second, the biological importance of enhancer clustering lies in its capacity to integrate cues and stimuli from multiple sources. For example, the efficient expression of the chemokine CCL20 requires the convergence of the transforming growth factor β (TGF-β) and interleukin-1β signalling pathways on an enhancer upstream of the *CCL20* promoter [117]. More interestingly, many of the extracellular signalling pathways important for ESC identity – such as leukaemia inhibitory factor (LIF), TGF-β and Wnt – converge on long stretches of enhancers along with OSN binding, to regulate target gene expression important for cell identity [49,108,118,119]. Furthermore, in a potential feed-forward mechanism, the expression of *Oct4* itself is regulated by a nearby enhancer also containing TFBSs for many of the TF effectors of the various signalling pathways [120]. Recent studies have also clearly demonstrated that multiple enhancers embedded within a cluster may operate in a partially redundant manner to fine tune gene expression [114] as well as enforce robustness in gene activity [115].

## Enhancer misregulation in human diseases: insights and avenues for intervention

Given the prominent role of enhancers and enhancer clusters in gene expression regulation, it is unsurprizing that aberrant enhancer function is involved in numerous diseases, as exemplified by the tremendous amount of mutations that have been identified at non-coding regulatory regions such as enhancers by genome-wide associated studies (GWAS) [86,87,108,121–123]. For example, single base pair point mutations have been described in the distal enhancers of *SNCA* and *PTF1A* gene, causal for sporadic Parkinson’s disease and pancreatic agenesis respectively [124,125].

Furthermore, both somatically acquired and lost super-enhancers have been identified in numerous cancers [108,112]. The finding that super-enhancers drive the expression of many oncogenes such as c*-Myc* has opened up novel transcription-based strategies to tackle human diseases via disruption of super-enhancer activity [126–128]. Apart from cancers, super-enhancers have been implicated in many complex human diseases such as Alzheimer’s disease, Type 1 diabetes and autoimmune disorders [108,112,129,130]. For example, reduced activity of super-enhancers, indicated by decreased H3K27ac enrichment, have also been found to down-regulate the expression of neuronal identity genes in the striatum of Huntington’s disease in mice [110].

## Enhancer function assessment: challenges ahead

As a large number of enhancers have been identified across different tissues and conditions [123,131,132], a pressing challenge is to functionalize these enhancers and to identify their cognate target genes and potential binding TF partners. Notably, not all identified enhancers are indispensable and a genome scale functional confirmation of enhancer function is necessary. The use of CRISPR-Cas9 genome editing technique will be a valuable tool to assess enhancer function, including GWAS risk variants that are located in enhancers [114,115]. For example, a recent study employed CRISPR-Cas9 to assess the function of the GWAS risk variants associated with Parkinson’s disease. In this case, the risk variants were located in a putative enhancer of the *SNCA* gene, edited into isogenic human pluripotent stem cells, and the impact of the mutations assessed as a function of neuronal differentiation [124].

Importantly, a key ingredient in functional verification of enhancers is the identification of target genes. Enhancers are frequently assigned to target genes that are linearly closest on the same chromosome [108,112,114]. Though it might be true in many cases that enhancers tend to regulate the expression of the nearest genes in *cis* [114], studies have shown that this might not always be accurate and thus enhancer–promoter interaction maps should provide valuable insights. For instance, by projecting SNPs on to enhancer–promoter interaction map, Won et al. [98] have shown that disease SNPs overlapping the enhancer regions and their nearest genes do not always interact. In another elegant study, Claussnitzer et al. [133] demonstrated that rs1421085, an obesity-associated SNP present in the first intron of the fat mass and obesity-associated (FTO) gene, was actually not affecting FTO expression, but instead of Iroquois homeobox 3 (*IRX3*) and Iroquois homeobox 5 (*IRX5*) through long-range interactions [133,134]. These studies highlight the importance of incorporating 3D genome information when assessing the role of non-coding variants in complex genetic diseases. Furthermore, due to the crucial roles of TFs in the establishment of enhancer–promoter interaction and tissue-specific gene expression, the genome scale identification of the potentially involved TFs is of extreme importance. One approach to achieve this is called the gene-centred yeast one hybrid assay which simultaneously detects the interaction between a pool of DNA regions and an array of TFs [135]. The finding that an enhancer region can bind to multiple proteins such as those encoded by paralogous genes, suggests that this approach, when integrated with tissue-specific expression profiles of TFs, could massively deepen our understanding on enhancer functions by interrogating their binding partners.

## Concluding remarks

In this review, we have established the importance of enhancers as a key integrating hub that synthesizes extrinsic and intrinsic signals, conveying the amalgamated information to promoters to shape the level and pattern of gene transcription. We believe that enhancer–promoter interaction maps provide an important context in assessing the consequences of non-coding genetic variations observed in disease states. Given that a huge number of non-coding sequence variants have been identified by multiple GWASs so far, and that the functional role of most of these non-coding variants remains largely unknown, we anticipate that chromatin interaction maps will aid in filling this knowledge gap.

## Abbreviations

BAF: barrier-to-autointegration factor
CCL20: chemokine (c-c motif) ligand 20
CFTR: cystic fibrosis transmembrane conductance regulator
CGN: cerebellar granule neuron
CREB: cAMP response element binging protein
CRISPR-Cas9: clustered regularly interspersed short palindromic repeats-CRISPR associated protein 9
CTCF: CCCTC-binding factor
DBD: DNA binding domain
EPHA4: EPH receptor A4
ERα: oestrogen receptor α
eRNA: enhancer RNA
ESC: embryonic stem cell
FoxA1: Forkhead Box A1
FTO: fat mass and obesity associated
GWAS: genome-wide associated study
H3K4me1: histone H3 lysine 4 monomethylation
H3K4me3: histone H3 lysine 4 trimethylation
H3K27ac: histone H3 lysine 27 acetylation
H3K27me3: histone H3 lysine 27 trimethylation
H3K36me3: histone H3 lysine 36 trimethylation
HNFa: hepatocyte nuclear factor alpha
IFN-β: interferon- β
IHH: indian hedgehog homolog
MED1: mediator subunit 1
NMDA: N-methyl-D-aspartate
OCT4: octamer-binding transcription factor 4
OSN: OCT4, SOX2 and NANOG
PAX3: paired box gene 3
PTF1A: pancreas specific transcription factor 1a
RNAPII: RNA polymerase II
SOX2: SRY (sex-determining region Y)-box 2
SP1: specificity protein 1
TAD: topologically associating domain
TEX10: testis expressed 10
TF: transcription factor
TFBS: transcription factor binding site
TGF-β: transforming growth factor β
TSS: transcription start site
WNT-6: wnt family member 6
ZIC: zinc finger in cerebellum
